# A Clinical Study on the Treatment of Multiple Radial Fractures with Embedded Wearable Device Holder and Absorption Bone Nail Combined with Decoction

This article has been retracted.

**DOI:** 10.1155/2021/6617823

**Published:** 2021-03-04

**Authors:** Zhilong Ren, Xiangyang Li

**Affiliations:** ^1^Department of Orthopedics 1, The First Hospital of Yulin, Yulin 719000, Shaanxi, China; ^2^Department of Bone and Joint, Baoji City Hospital of Traditional Chinese Medicine, Baoji 721001, Shaanxi, China

## Abstract

Multiple radial fractures have brought great pain to the patients, and the treatment takes a long time and the effect is slow, which seriously affects people's production and life. Traditional conservative treatment methods are mostly used for radius fractures. However, with the development of science and technology of the times, the level of medical treatment is also constantly improving. For radius fractures, the embedded wearable device fixation frame absorption bone nail treatment method has attracted attention. In order to study whether the embedded wearable device fixation frame can treat radius fractures, this article conducted a related survey of radius fracture patients in a hospital in a certain city, reviewed related literature, conducted interviews with professionals and so forth, and collected relevant information. A case template was constructed, and a clinical research model was created using a comprehensive quantitative and qualitative analysis method. The results of the study found that using the research embedded wearable device fixation frame to treat radius fractures with absorption bone nails can achieve good results, and its healing efficiency is about 20% faster than conservative treatment. With decoction, its treatment efficiency can be improved; and the prognostic treatment of the decoction can reduce the complications of the patient's treatment by about 13%. This shows that the embedded wearable device holder absorption bone nail combined with decoction can play an important role in the treatment of multiple radius fractures.

## 1. Introduction

The radius is an important part of the elbow joint. The radius and the head of the humerus form the humeral joint, and the small sigmoid notch between the inner radius and the ulna forms the proximal radioulnar joint. The radius is a vulnerable structure. After elbow joint trauma, it is easy to be complicated by heterotopic ossification and poor healing is easy to be complicated by joint stiffness. Therefore, if the radius fracture is not handled properly, the function of the elbow joint will be severely impaired [1]. Radial head longitudinal conduction violence is a common cause of radius fractures. When a person accidentally falls, the palm of the hand touches the ground, the elbow is in an extended position, the upper limb is abducted, and, due to the existence of the lifting angle, the elbow is extremely valgus and the elbow is affected. The strong longitudinal stress caused the radial head to hit the humeral head and caused the former to fracture [2]. Distal radius fractures mostly occur in middle-aged and elderly women. Many patients have osteoporosis. Most of the distal radius fractures are caused by low-energy traumas such as falls, while joint fractures are mostly caused by high-energy and more violent traumas [3].

For closed distal radius fractures, there have been a large number of reports in the literature. There are many types of surgical methods, including volar approach plate screw internal fixation, dorsal approach plate screw internal fixation, external fixation bracket, intramedullary nail, percutaneous Kirschner wire fixation, wrist arthroscopy, and wrist joint replacement surgery; internal fixation with steel plate and external fixation have their own advantages. The choice of surgical method mainly depends on the type of fracture, whether there is nerve and tendon damage, the age of the patient, the underlying disease, general condition, and the patient's wishes; compared with closed distal radius fractures, open distal radius fractures are more violent, with more damage to soft tissues, tendons, nerves, and so forth, and fractures do not heal. Complications such as postoperative infection and joint stiffness are more common. Therefore, some literature reports that the treatment effect of open distal radius fractures is not as good as closed distal radius fractures [4]. Many experts at home and abroad have studied radius fractures.

In order to study the manual reduction of radius fractures in children, Cha Tianwen divided the children into three groups through statistics of children's radius fractures that occurred within two years and conducted relevant statistics on the treatment methods and curative effects of their fractures. He concluded that children radius fractures can be treated by manual reduction and surgery, and both have continuous effects. However, in terms of clinical effects, the healing rate of surgical treatment is higher than that of manual compound [5]; Li believes that radius fractures can be treated by high-frequency ultrasound. Through the statistics of radius fracture cases admitted to the Affiliated Hospital of Chengde Medical College, a controlled experiment was established to target and guide the fracture site by using high-frequency ultrasound on patients with radius fractures, so that the fracture site could be fixed with internal nails and the fracture site reduction treatment [6]; Ou believes that traditional Chinese medicine has a certain effect on the prognosis of radius fractures. It uses traditional Chinese medicine fumigation to perform prognostic treatment for patients with radius fractures that have been treated. By comparing the recovery conditions of untreated patients, such as joint flexion and fracture site parameters, experimental results show that traditional Chinese medicine fumigation can significantly improve patients' blood flow indicators, reduce serum levels, and benefit the prognostic healing of patients with radius fractures [7]. These studies provide a certain reference value for our experiments, but, due to insufficient experimental samples and unclear experimental methods, their conclusions are somewhat sloppy and unconvincing.

In this paper, by establishing a calculation model for radius fracture healing, the therapeutic effect of the embedded wearable device fixation frame absorption bone nail combined with decoction is compared with other fracture treatment methods in all aspects to test whether it can play a role in radius fractures. Through the collection of relevant experimental data, a more detailed multilevel analysis of the comparison results of the experimental data finally concluded that, based on the test of patients and experts, the experimental conclusions show that the embedded wearable device holder absorbs bone nails and soup drug therapy has high practical value for the treatment of radius fractures.

## 2. Embedded Wearable Device Fixing Frame Absorbs Bone Nails and Decoction Treatment Method

### 2.1. Radius Fractures and Treatment Methods

Due to the development of modern society and economy, transportation and industry are becoming more developed, and high-energy damage is increasing. Simple radial fractures are rare, and other parts of the elbow joint are easily damaged at the same time. At the same time, due to the improvement of human life quality expectations, the requirements for the recovery of the elbow joint function after injury are getting higher and higher, so the requirements for the treatment and rehabilitation of the radius trauma are also getting higher and higher, but the elbow joint is prone to ankylosis and heterotopic ossification is prone to occur, so orthopedic surgeons have also put forward higher requirements [8]. The development of treatment concepts in elbow joint surgery in China is lagging behind that of European and American countries. Therefore, orthopedic surgeons in China should improve their professional skills in elbow joint surgery.

Radius replacement can prevent bone from growing from the upper short end of the radius and prevent the formation of myositis ossificans. In the early stage of the replacement surgery, the radial support force can be restored and the elbow joint valgus can be prevented. It can maintain the structural stability of the elbow joint, thereby maintaining the physiological tension of the ligaments, which is beneficial to the repair of the ligaments around the elbow joint, better maintains the stability of the elbow joint, and reduces the radial movement caused by the simple radius resection, which causes the wrist symptoms such as joint pain [9].

The role of the radial head in the forearm is mainly reflected in rotation and lateral support. It is an important structure for elbow joint flexion and extension and rotation. The lateral stability mechanism of the elbow joint requires the integrity of the medial collateral ligament and the height of the radial head to be maintained. The integrity of the bony structure is very important for the stability of the elbow joint function [10]. Adults with strong muscle strength, unstable fracture ends, limb lengthening, and joint deformity correction usually require higher fixation strength. Thick needles should be appropriately selected and the number of bones should be increased. The diameter of the bone meal should be determined according to the size and thickness of the patient's bone. When the soft tissue is thick, half needles should be used; when soft tissue defects, ulcers and burns with infection, fine needles, and half needles are selected locally, and needles are added at the remote site; for soft tissues for contractures and scars, the amount of bones should be increased and thicker bones should be used [11].

### 2.2. Embedded Fixing Frame

After the orthopedic brace for external fixation is installed, the length of each connecting rod can be read through the scale marks on the connecting rod. It is necessary to determine the spatial pose of the current fixing ring through the length of the connecting rod and adjust the length of the six connecting rods. The posture of the fixed ring can achieve restoration and deformity correction of fractures [12].

According to the simplified table-type six-degree-of-freedom parallel mechanism based on the orthopedic bracket for external fixation, the upper platform pose is calculated from the link length, and the positive kinematics analysis of the parallel mechanism is performed. Due to the complexity of the parallel mechanism and the difficulty of position forwarding, the commonly used calculation methods include analytical and numerical methods [13]. The numerical method is to establish a set of nonlinear equations and use an approximation method to solve the nonlinear equations, thereby calculating the pose of the moving platform corresponding to the length of the input link. In order to quickly calculate the position and posture of the fixed ring relative to the lower fixed ring of the fixed bracket, this paper uses a numerical method to perform a forward position solution of the table-type six-degree-of-freedom parallel mechanism. Based on the inverse position of the parallel mechanism, it is easy to find the position and iterative calculation of the connecting rod length. The pose of the moving platform is constantly modified, and the pose of the moving platform under a certain rod length is approximately solved [14]. The manufacturing method of the fixing frame is shown in Figure 1.

Many scholars have made various improvements to the external fixator according to the actual clinical situation. In the process of improvement, a mechanical environment conducive to fracture healing must be established. The external fixator has good stability, flexible structure, easy adjustment, less tissue damage, and so forth. In the actual orthopedic process, when the upper and lower ring models are certain, due to the single structure of the current fixation frame and lack of flexibility, the support rod may interfere with the limbs. Especially for open fractures, the soft tissue damage is serious, making the correction impossible. He needs to reclamp, bring pain to the patient, but also increase the risk of surgery. If the space between the connecting rod and the affected area is small, it is not conducive to postoperative dressing change or secondary debridement and secondary repair treatment [15]. If you choose a larger fixing ring, the structural space of the fixing frame will be relatively large, the length of the steel needle required for bone fixation will increase, and the overall structural stability of the fixing frame will decrease. It is necessary to increase the number of needles or the diameter of the steel needle to improve the rigidity of the fixing, which increases the chance of needle tract infection [16]. At the same time, the frame installed on the patient's limb is too large, and the weight of the fixing frame also increases, which affects the patient's rehabilitation training.

The stability of the fixation is mainly determined by the spatial geometry formed by the steel needle, the fixing clip, and the connecting rod as well as the material properties of the steel needle, the fixing clip, and the connecting rod [17]. Therefore, the bone external fixator is designed to meet the needs of multidirectional needle penetration. During the fracture healing process, its stability can be adjusted appropriately according to the rehabilitation situation, and materials with appropriate elastic modulus and specific gravity can be selected.

The bone external fixator should be simple to operate and easy to assemble and disassemble, can have the functions of restoration and fixation and adjustability, and can appropriately adjust the fracture fixation stiffness after the operation [18]. After the fracture is fixed, there is enough space left between the fixator and the affected area, which is easy for postoperative soft tissue repair and wound dressing or second postoperative debridement. We have the following formula:

(1) $$\begin{array}{c} r=\frac{\text{pnd}}{\lambda },\\ N=0.25r^{0.8}{\mathrm{Pr}}^{0.4},\\ \frac{\alpha *d}{\sigma }=0.25{\left(\frac{d*r*p}{\kappa }\right)}^{0.8}{\left(\frac{c*u}{\sigma }\right)}^{0.4}. \end{array}$$

After simplifying the above formula, we get

(2) $$\begin{array}{c} \alpha =\frac{2.057f*{\left(v*p\right)}^{0.8}}{d^{0.2}},\\ \;\sum_{n=1}^{i}\left(\vartheta r_{n}*w_{n}r_{n}+\vartheta \mu_{n}j_{n}\mu_{n}\right)-\sum_{j=1}^{i}\vartheta \theta_{n}\nu_{n}-\vartheta r_{i}*S_{i}=Q,\\ \vartheta =\frac{6}{5\left(a_{i}+a_{j}\right)}{\left[\frac{r_{i}r_{j}}{r_{i}+r_{j}}\right]}^{\left(1/2\right)},\\ a_{n}=\frac{1-t_{n}^{2}}{S_{n}},\;\left(n=i,j\right). \end{array}$$

For cases with bone defects, microplates can also be used after local bone grafting. However, it is necessary to understand that the internal fixation with steel plate is traumatic, the proximal radius is exposed, the dissection area is increased, the blood supply is increased, the possibility of bone nonunion and radial head necrosis is increased, and the fixation site can only be placed in a safe area. Therefore, steel plate internal fixation should be used in cases with severe injuries such as those mentioned above. At the same time, it is necessary to explain the possibility of the above complications to the patient and family members. During the operation, the operation is gentle and the tissue around the fracture should be protected to prevent further damage to the blood supply [19]. The effects of metal nails and steel plates are different. The poor effect of steel plate internal fixation in some documents may be considered. Possible reasons are as follows: 1. Incorrect choice of indications, such as comminuted fracture of the radial head, forcibly uses internal fixation instead of choosing small radius. Head resection or replacement of the radial head leads to poor functional recovery, but this is often difficult to define. 2. The microplate internal fixation itself is used in patients with severe injuries, and the prognosis itself is poor. There is no statistical difference between bone gluten fixation and steel plate fixation in the evaluation indexes of joint function and fracture recovery time. Therefore, the correct selection of indications, bone fixation or plate fixation, has a great impact on fracture healing and functional recovery.

### 2.3. Absorbable Bone Nail

With the development of biodegradable materials, the technology of absorbable screws has developed and the use has increased. The absorbable screw can finally be degraded into carbon dioxide and water in the body, and finally there is no object left. Animal experiments and long-term clinical experiments have proved the safety of the absorbable screw. Absorbable screws have good flexibility and strong shear resistance, and the strength can reach the hardness of cortical bone. The initial bending strength can be maintained for more than 4 months after being placed in the human body. The healing time of patients with absorbable screws is 13.38 ± 2.43. Therefore, the strength and degradation time of the absorbable screw in the body meet the needs of healing [20]. The absorbable screw has the ability of lateral expansion, which can make the fixation more secure. In the process of fracture healing, due to the absorption of the absorbable screw, the stress shielding of the fracture site will be gradually reduced compared with the metal nail, which can avoid local osteoporosis. However, it should be noted that the joint cavity and interstitial space basically have no absorption or degradation ability for the absorbable screw material. For example, because the screw is not completely absorbed, foreign bodies in the joint cavity or surrounding tissue will be formed, which will affect the recovery of joint function and even require surgical removal. Pay attention to the countersunk treatment of the screw, so that the screw completely enters the bone tissue and can be trimmed appropriately if necessary [21].

Regarding the general use process of the orthopedic stent for external bone fixation, the surgeon diagnoses and treats the wound of the patient, selects the appropriate needle insertion position, and fixes the two appropriate size fixing rings to the appropriate bone end of the fracture through the fixing clip and the steel pin. The connecting piece is installed on the fixed ring. The doctor can choose the flat connecting piece or the Z-shaped connecting piece according to the actual situation of the patient. The connecting piece can be installed on the remaining mounting holes of the fixed ring. The installation position can be evenly distributed or installed close to the actual situation. Hole, compared with Taylor space bracket, has greater flexibility [22]. Choose six connecting rods of appropriate length and adjustment range, install them on the connecting pieces of the upper and lower fixing rings in a certain order, or directly install them on the remaining holes of the fixing ring. Input the selected component information into the computer program, measure the corresponding parameters on the X-ray film through human-computer interaction, and finally calculate the deformity correction parameters and formulate the orthopedic prescription to achieve fracture reduction and deformity correction [23].

After open reduction and internal fixation, the radial head can be preserved, so the shape and length of the radial head can be restored at the same time. However, internal fixation treatment requires a longer external fixation time, and a longer postoperative external fixation time will cause joint stiffness, secondary trauma, and other unfavorable factors that affect the recovery of elbow joint function. Most scholars believe that the effect of radial head replacement is better than radial head open reduction and internal fixation, and the incidence of complications is also lower than that of radial head open reduction and internal fixation [24]. However, considering that there is no long-term follow-up effect for radial head replacement and, at the same time, there are the aforementioned complications and the incidence of some complications gradually increases with the prolonged treatment time, the choice of radial head replacement needs to be cautious and try to choose internal fixation. But, for radial head fractures that cannot be completely reduced, especially if there are more than three fractures, the effect of internal fixation is often poor, and the recovery of elbow joint function may be poor [25]. We have the following equation:

(3) $$\begin{array}{c} U_{a}=p*b\frac{j}{i}*c. \end{array}$$

We ensure the objectivity of the evaluation results by calculating the weights of attributes:

(4) $$\begin{array}{c} p=\frac{1}{\sin x}\sum_{n=1}^{1}f_{nm}*\;\ln\;f_{nm},\\ j=\frac{1-i}{y-\sum_{m=1}^{m}t}+\frac{1}{1+d\left(r_{x},uq\right)},\\ f_{mn}=\frac{z_{nm}}{\sum_{n=1}^{x}z_{nm}},\\ \overset{x}{\underset{m=1}{\sum }}w_{m}=1. \end{array}$$

Set objective weight:

(5) $$\begin{array}{c} d=\sqrt{\sum_{m=1}^{x}w_{n}*{\left(r_{nm}-uq_{m}\right)}^{2}},\\ d_{n}=\frac{1}{1+d\left(r_{n},uq\right)},\\ Q_{\delta }=\left\{r_{n}\left|d\;\cos\left(r_{n},uq\right)\right|\geq \delta \right\},\\ \kappa =\frac{\sum \left(q_{rp,rpn}-q_{rpm}\right)\left(q_{uq,uqn}-q_{uq}\right)}{\sum_{n=1}^{n}{\left(q_{r}-q_{uq}\right)}^{2}\sqrt{\sum {\left(q_{uq,uqm}-q_{uq}\right)}^{2}}}. \end{array}$$

### 2.4. Prognostic Treatment

Incision problems are the most common postoperative complications of fractures. Most of the incision skin necrosis or incision infection injury to the operation time is closely related to the postoperative incision complications. Appropriate operation timing has a greater impact on the postoperative prognosis of radius fractures. However, there is a lot of controversy over the most appropriate time to perform surgery. Some scholars believe that surgery should be performed after the soft tissue condition improves, which can help soft tissue swelling and reduce the rate of skin flap necrosis. Some others believe that surgery should be performed as soon as possible after injury. Treatment can reduce the pressure of swelling on surrounding soft tissues and reduce the incidence of complications after soft tissue surgery.

In order to ensure that early related joint function exercises can be carried out after radius fractures and to reduce related postoperative complications, it is necessary to ensure the stability of internal fixators. In addition to fracture classification, the choice of treatment options for radius fractures should also consider age and fracture damage and whether it is combined with other related comorbidities. For young patients, conservative treatment and surgical treatment can achieve better results. For elderly patients, it is recommended that conservative treatment of open fractures requires a first stage of debridement and drainage. After the wound is closed, there is no obvious second-stage surgical treatment after infection signs. With the further analysis of the treatment of radius fractures in terms of biomechanics, it is found that not only is a good prognosis of radius fractures related to the type of fracture but also the reduction of the posterior articular surface also plays an important role.

Due to the poor blood supply of the soft tissue around the radius and the large impact on the surrounding tissues during fracture, postoperative complications are mostly divided into early complications and long-term complications. The former mainly include incision skin necrosis and incision infection, while the latter mainly include fracture malunion and traumatic arthritis, which seriously affect the life of patients. Therefore, in the surgical treatment of radius fractures, not only should the relevant preoperative preparations be made and should the correct surgical method and surgical approach be selected, but also the anatomical reduction must be restored Reduce surgical trauma, thereby improving surgical efficacy and alleviating patient suffering. After treatment, relevant prognostic treatment should also be done to prevent various complications.

According to related studies, traditional Chinese medicine fumigation can improve fractures. This article uses relevant Chinese medicine decoctions for the prognosis of the treated patients and performs relevant nursing care to avoid related complications. The treatment of radius fractures has the same treatment principle, that is, to restore the anatomical reduction of the radius as much as possible, and prevention and treatment. Postcomplications restore the function of the affected limb as much as possible. With the continuous improvement of medical standards and the deepening of understanding of radius fractures, our treatment of radius fractures and the prevention of postfracture complications will surely reach a new height.

## 3. Experimental Method of Radius Fracture

### 3.1. Experimental Purpose

This article is based on the theoretical results of the treatment of radius fractures, draws on the domestic and foreign theoretical research results, and uses literature, comparative research, mathematical statistics, logical analysis, and other methods to absorb bone nails from the embedded wearable device fixed frame and decoction to treat multiple cases. Indepth analysis of radial fractures, etc., to study its application methods and characteristics.

### 3.2. Experimental Judgment and Prognostic Treatment

The entropy method is a relatively objective evaluation index weight assignment method, which can effectively avoid the subjectivity of artificial scoring and has high accuracy. But, at the same time, this study also realizes that the entropy method has the defect that it cannot directly reflect the knowledge, opinions, and empirical judgments of experts and scholars, and the weighted results obtained may be contrary to reality. Therefore, this article uses a combination of analytic hierarchy process and entropy method to determine the weight coefficient of each evaluation index of regional higher education.

As regards comprehensive quantitative and qualitative analysis methods, quantitative analysis is to analyze the data of the problem, using the intuitive and clear essence of mathematics to reflect the existence of the problem; qualitative analysis is to collect, read, organize, and systematically analyze the relevant theoretical results. Some standards cannot be directly analyzed in a quantitative way but can only be evaluated using a qualitative analysis method. The assessment standard system is constructed using a combination of quantitative and qualitative analysis methods, and formulas related to standard calculations are also given.

Within 24 hours after surgery, he was given a first-generation cephalosporin intravenous infusion to prevent infection, dehydration, swelling, and pain relief, as we ll as oral indomethacin to prevent heterotopic ossification. Except for patients with embedded fixation stents, all other patients received external plaster fixation. Begin to move the affected limb after the operation, and guide the isometric contraction training of the biceps and triceps. In the first 1–3 weeks after the operation, the plaster cast was removed and the patient was instructed to perform forearm rotation and active elbow joint flexion and extension exercises. The sutures were removed two weeks after the operation, and the outpatient review was conducted in January, February, and March after the operation to guide functional exercise and observe the patient's recovery. During the exercise, pay attention to avoid elbow extension.

### 3.3. Data Sources

This article uses embedded fixation, bone nails, radius fractures, and so forth as keywords, and the start and end years are set to 2015–2019. The network platforms such as CNKI and Baidu are used to find relevant literature, and the collected data are classified and sorted to obtain. There are 167 Chinese and foreign academic papers, 29 academic books, 34 newspapers and online materials, and 15 doctoral and Master's theses related to this research. At the same time, it collects patients and doctors' opinions on embedded wearable devices through questionnaire surveys and field interviews. There are also views on the treatment of multiple radius fractures with fixed frame absorption bone nail and decoction.

## 4. Experimental Analysis of Multiple Radial Fractures

### 4.1. Population Distribution of Radius Fractures

We collected statistics on the population who had undergone radial fracture treatment in the city hospital and classified them according to factors such as age and gender. We hope to find out the characteristics and laws of radius fractures. The specific data of the patients are shown in Table 1.

According to Figures 2 and 3, we can see that the degree of radius fractures varies between different ages. The population of radius fractures is mainly distributed among young and middle-aged, that is, below 45 years, a total of about 540 people, accounting for this survey population. In people over 60 years of age, the number of radius fractures is about 150, accounting for about 17% of the total number. This shows that radius fractures will occur in young and middle-aged people, and related treatment methods should also be tilted to the side. We also investigated the gender of the population, as shown in Table 2 and Figure 4.

### 4.2. Treatment of Radius Fractures

For radius fractures, the current treatment methods include external fixation, absorptive bone nails, conservative treatment, embedded fixation, and the embedded wearable device fixation used in this article. The method of absorbing bone nails and medicines is used in this article. We make statistics on the current treatment population. The detailed data are shown in Table 3.

From Figure 5, we can see that, for most patients, it is not the first choice to use the embedded wearable device holder to absorb bone nails and medicines for treatment. This is because this method requires more steps. For people with mild radius fractures, they are more inclined to choose conservative treatment or other treatment methods. However, with the development of time, the embedded wearable device fixation frame absorption bone nail combined with pharmaceutical treatment has been more and more accepted by people. We have calculated the data from 2010 to 2019, as shown in Table 4.

It can be seen from Figure 6 that, over time, the treatment of radius fractures has also undergone certain changes. Although conservative treatment is still the first choice for the treatment of radius fractures according to patients, in recent years, the use of embedded wearable device holders to absorb bone nails and drugs for treatment has been recognized and tried by more and more people.

### 4.3. Effects of Different Treatment Methods

For multiple radius fractures, the treatment effect is the most concerned issue for patients. We have carried out quantitative calculations on different methods of treatment through the calculation model mentioned in the article and carried out relevant statistics. According to the calculation results, the final value is above 0.8 for excellent healing effect, and the value is above 0.5 for passing. The specific statistical results are shown in Table 5.

It can be seen from Figure 7 that the methods in this article basically scored more than a few and scored more than 0.8 in temperature and painlessness. Compared with other methods, in bone absorption through the embedded wearable device holder, not only can the nail compound with the medicine remain stable during the treatment process, but also it performs extremely well in other aspects. The prognostic treatment of radius fractures is also extremely important. In this regard, we have counted several important indicators of fracture prognosis, which are shown in Figure 8.

We can see from Figure 8 that, in terms of prognosis, the use of embedded wearable device holders to absorb bone nails and drugs to treat radius fractures also has many advantages in prognostic treatment, and its score is basically maintained above good. Although other methods have their own advantages, in general, the embedded wearable device holder to absorb bone nails and drugs can play an important role in treatment and prognosis.

## 5. Conclusions

Embedded wearable device fixation technology is to use steel needles or steel nails to penetrate the bone structure through the skin and soft tissue on the bone segments at both ends of the fracture and then use connecting rods and fixation clips to connect and fix the external fixation on the external fixation frame. It can achieve the purpose of good reduction at both ends of the fracture and local damage control.

Radius is damaged due to elbow trauma, and healing is often delayed, leading to poor recovery of elbow joint function. At the same time, there is also the possibility of fracture nonunion or malunion, especially in cases with many fractures and large trauma, which may require a second treatment, which may cause damage to the elbow joint and increase the incidence of elbow joint movement restriction. The embedded wearable device holder absorbs bone nails to prevent bone from growing out of the short end of the upper end of the radius and can prevent the formation of ossifying myositis. It can better restore radial support and resist elbow valgus. It can maintain the structural stability of the elbow joint, thereby maintaining the physiological tension of the ligaments, which is beneficial to the repair of the ligaments around the elbow joint, better maintains the stability of the elbow joint, and reduces the upward movement of the radius caused by simple radius fractures and thus the wrist joint pain and other symptoms.

In recent years, the development of the Internet has been changing with each passing day, and China has also accelerated its policy support for independent innovation and localization of medical devices, especially the concept of “Internet + medical treatment” proposed to carry out human bone orthopedic devices and fracture corrections. Algorithm development is of great significance for promoting the development and progress of bone orthopedic medical devices in China.

## Figures and Tables

**Figure 1:** Embedded fixing frame production.

**Figure 2:** Population distribution.

**Figure 3:** Age distribution of radius fractures.

**Figure 4:** Gender population distribution.

**Figure 5:** Radius fracture treatment.

**Figure 6:** The difference in treatment in different years.

**Figure 7:** Treatment effect of different methods.

**Figure 8:** Prognostic treatment score.

**Table 1:** Distribution of radius fracture population.

Age	Minor fracture	General fracture	Severe fracture	Very severe fracture	Fractured bone
0–12	3	8	11	7	8
13–26	66	88	31	47	18
27–45	57	61	99	36	26
46–60	32	91	87	53	13
Over 60	27	42	51	21	9

**Table 2:** Gender distribution.

	Minor fracture	General fracture	Severe fracture	Very severe fracture	Fractured bone
Male	103	213	195	109	49
Female	82	87	84	55	25

**Table 3:** Difference in treatment.

	Minor fracture	General fracture	Severe fracture	Very severe fracture	Fractured bone
External fixator	3	29	47	31	21
Absorbing bone nail	1	21	51	26	13
Conservative treatment	26	54	63	47	19
Embedded fixation	5	19	27	29	15
Method of this article	2	36	19	26	12

**Table 4:** Difference in treatment.

	2010	2011	2012	2013	2014	2015	2016	2017	2018	2019
External fixator	37	44	49	66	57	63	75	51	47	42
Absorbing bone nail	19	21	27	33	51	47	41	39	46	41
Conservative treatment	67	72	79	69	88	109	97	89	81	76
Embedded fixation	29	36	33	42	39	33	45	47	56	55
Method of this article	1	3	9	15	13	17	23	26	33	37

**Table 5:** Treatment effect of radius fracture.

	Stability	Flexibility	Bone setting effect	Recovery effect	Pain	Sequelae
External fixator	0.537	0.887	0.528	0.718	0.642	0.516
Absorbing bone nail	0.431	0.573	0.431	0.752	0.669	0.678
Conservative treatment	0.479	0.526	0.888	0.697	0.477	0.617
Embedded fixation	0.539	0.643	0.542	0.573	0.681	0.854
Method of this article	0.879	0.735	0.779	0.697	0.813	0.725

## Data Availability

No data were used to support this study.
